# Posterior Mitral Leaflet Prolapse and Subsequent Mitral Valve Endocarditis Complicated With Anterior Leaflet Perforation

**DOI:** 10.7759/cureus.36315

**Published:** 2023-03-17

**Authors:** Hideki Sasaki, Yukihide Numata, Jien Saito, Shinji Kamiya, Miki Asano

**Affiliations:** 1 Cardiovascular Surgery, Nagoya City University East Medical Center, Nagoya, JPN

**Keywords:** bacterial biofilm, epilepsy, brain infarction, mitral valve perforation, mitral valve regurgitation, infective endocarditis

## Abstract

A 68-year-old male presented with a two-week history of fever, and further investigations revealed mitral valve endocarditis caused by *Staphylococcus epidermidis*, with associated severe mitral regurgitation (MR). The patient was referred for mitral valve surgery but developed new neurological symptoms two days before the operation, which were diagnosed as symptomatic epilepsy. During surgery, kissing lesions were found on the posterior mitral leaflet (PML), which were not detected on preoperative transesophageal echocardiography (TEE). Mitral valve repair was completed using autologous pericardium. The current case highlights the importance of careful examination of leaflets during surgery and not relying solely on preoperative imaging to detect all lesions. It is essential to promptly diagnose and treat infective endocarditis to prevent further complications and ensure successful outcomes.

## Introduction

Infective endocarditis is a life-threatening disease, and its symptoms can vary depending on specific conditions [1-3]. Although antibiotics are the first-line treatment, subsequent complications such as embolism, heart failure, and septicemia can occur. Brain infarction is one of the most serious complications caused by vegetation [4-6]. The related neurological symptoms can present difficult problems for physicians to diagnose and treat, as they can be caused by a variety of underlying conditions. We present a patient whose mitral valve was destroyed by *Staphylococcus epidermidis* and who presented new neurological symptoms immediately before surgery.

## Case presentation

A 68-year-old male presented to a family physician complaining of two weeks of fever. The patient has been diagnosed with severe mitral regurgitation (MR) at another clinic three years ago. Despite the physician’s advice for the patient to visit a cardiology clinic, he did not accept it. Transthoracic echocardiography (TTE) revealed large vegetation, perforation of the anterior mitral leaflet (AML), and prolapse of the posterior mitral leaflet (PML). Blood culture was positive for *Staphylococcus epidermidis*. Head computed tomography was performed for screening, which revealed an old brain infarction at the right frontal lobe. Transesophageal echocardiography (TEE) demonstrated vegetation and the perforation, 6.5 mm in diameter at the A2 segment of the AML with prolapsed P1 of the PML resulting in severe MR (Figure 1 and Figure 2).

**Figure 1:** Preoperative transesophageal echocardiography Preoperative transesophageal echocardiography showing vegetation on the anterior mitral leaflet and prolapsed P1 of the posterior mitral leaflet

**Figure 2:** Preoperative transesophageal echocardiography Preoperative transesophageal echocardiography showing vegetation and perforation (✜) of the anterior mitral leaflet LV: left ventricle, LA: left atrium, Ao: aorta

Cefazoline was administered empirically. The patient was referred to the cardiovascular department, and mitral valve surgery was planned. However, the patient presented with conjugate deviation, left lower limb weakness, and consciousness disturbance two days before surgery. The results of the blood gas analysis indicate the presence of acidemia, as evidenced by a pH value of 7.219, a low bicarbonate concentration of 14 mmol/L, and a negative base excess (BE) of -12.4 mmol/L. Furthermore, the lactate level was found to be elevated at 9.1 mmol/L, suggesting a possible underlying metabolic disturbance. Head magnetic resonance imaging (MRI) revealed no new lesion, and magnetic resonance angiography (MRA) showed no occlusion of the cerebral artery (Figure 3). The patient was referred to a neurologist and was diagnosed with symptomatic epilepsy associated with the old brain infarction at the right frontal lobe. Levetiracetam was prescribed by the neurologist.

**Figure 3:** Head magnetic resonance angiography Head magnetic resonance angiography showing no occlusion of the cerebral artery

The operation was performed two days later as planned. Cardiopulmonary bypass (CPB) was established with ascending aortic perfusion and vena cava drainage. After opening the left atrium (LA), the mitral valve was inspected. Large vegetation and perforation were found at the A2 of the AML (Figure 4). The defect became 15 × 18 mm in its diameter after the radical removal of the vegetation and edematous tissue. The distance from the edge of the defect to the strut chordae was about 5 mm.

**Figure 4:** Intraoperative findings Vegetation on the anterior mitral leaflet

The autologous pericardium was harvested and trimmed to 25 × 28 mm. It was sutured to the defect using a 5-0 monofilament suture. A saline test revealed leakage from two points, one is from the prolapsed P1 and the other is from the indentation between P1 and P2 (Figure 5). The former was repaired using the folding plasty technique with two pairs of 5-0 monofilament sutures. The latter was repaired by suturing P1 and P2. A prosthetic ring (Carpentier-Edwards Physio II ring, Edwards Lifesciences, Irvine, CA, USA) was attached to the mitral annulus (Figure 6). The saline test revealed no MR. The patient was successfully weaned from CPB. Levetiracetam was restarted from postoperative day 1, and no epilepsy occurred. Antibiotic treatment was continued for six weeks, and the patient was discharged without complications.

**Figure 5:** Schematic drawing of mitral valve lesions Multiple lesions associated with vegetation, perforation on A2, prolapsed P1, and cleft between P1 and P2

**Figure 6:** Completion of mitral valve repair Mitral valve repair using autologous pericardium and annuloplasty ring; prolapsed P1 folded using monofilament sutures

## Discussion

*Staphylococcus epidermidis* is a gram-positive bacterium found in the skin and nasal cavity. Although it is generally not harmful, it can pose a risk for patients who are in a compromised condition such as those taking immunosuppressive drugs and have prostheses such as catheters and medical devices in the body [1,7]. In addition, a patient whose heart valve is regurgitant and stenotic or who has congenital heart defects is considered at high risk for infective endocarditis [1]. While timely surgical intervention can improve outcomes [5], neurological complications have a negative impact on prognosis [8,9].

The most concerning problem in the current case was neurological symptoms that occurred two days before surgery. During the patient examination, we suspected that the new brain infarction was caused by the vegetation. However, head magnetic resonance imaging (MRI) revealed neither cerebral artery occlusion findings nor cerebral hemorrhage. The patient was referred to the neurologist, and the diagnosis was symptomatic epilepsy attributed to the old brain infarction at the right frontal lobe.

Regarding the localization of affected lesions on the mitral valve, transesophageal echocardiography (TEE) plays an important role. However, it is important for surgeons to keep in mind that preoperative TEE may not detect all lesions. We found regurgitation from the cleft between P1 and P2 during the saline test that had not been detected on preoperative TEE. It would be necessary for surgeons not only to consider possible lesions preoperatively but also not to overlook unexpected lesions during operation. Although the lesion was restricted to the clear zone, the edge of the perforation was close to strut chordae, which is the most important subvalvular apparatus. If the suture needle catches it, the strut chordae will be shortened, and the anterior leaflet would fall into the left ventricle, which leads to severe MR. We prefer to use a 5-0 monofilament suture in suturing the pericardium to the leaflet. As the leaflet is thin and slightly edematous in acute IE, a small needle is better. Following pericardial patch repair in A2, the saline test showed regurgitation from two points. Although we knew the presence of prolapsed P1 preoperatively on TEE, indentation became visible by saline test and was repaired with P1-P2 closure using a 5-0 monofilament suture. Surgeons should always consider the presence of undetected accessory lesions during surgery.

In examining the valve, several kissing lesions were found on P2. We suspect that the vegetation on A2 contacted the PML, resulting in a new lesion on P2. They formed bacterial biofilm on the leaflet surface. A biofilm is a surface-attached microcolony of microbes encased in a self-produced matrix of extracellular polymeric substances acting as a protective slime layer [10]. After removing the biofilm with a suction device carefully, the surface became clear, and it turned out that the valve was not destroyed by the microbe. We thought that antibiotics would work more effectively by removing the biofilm. However, excessive curettage can cause unnecessary injury to the endothelium, and the lamina fibrosa would be exposed, which can lead to perforation. When the biofilm is misdiagnosed as valve destruction, it would be resected, and the defect must be reconstructed. It makes the operative procedure unnecessarily complicated. It is essential for surgeons to assess the lesions precisely.

In summary, the current case emphasizes the importance of a thorough preoperative evaluation, including TEE and blood cultures, to identify any vegetation or infections. Additionally, surgeons should carefully inspect the leaflets during surgery to identify any undetected lesions.

## Conclusions

It is crucial not to make a hasty diagnosis without appropriate diagnostic tests such as an MRI when encountering a patient with neurological symptoms and vegetation on the valve.

When inspecting an infected mitral valve, it is important for surgeons to perform a thorough examination of all leaflets and subvalvular apparatus to detect any accessory lesions that may not have been detected on preoperative TEE. Surgeons should also be aware of the concept of bacterial biofilm, which is a protective layer that forms around bacteria and can make them more resistant to antibiotics. Surgeons should be able to distinguish between a destructed valve and a biofilm, as this can affect the choice of surgical approach and postoperative management.
